The article "Rituximab-conjugated, doxorubicin-loaded microbubbles as a theranostic modality in B-cell lymphoma" was retracted in 2017. Reason: errors in the data.

# Rituximab-conjugated, doxorubicin-loaded microbubbles as a theranostic modality in B-cell lymphoma

**DOI:** 10.18632/oncotarget.13587

**Published:** 2016-11-25

**Authors:** Shoubing Zhou, Xiu Zhang, Cailian Wang

**Affiliations:** ^1^ Department of Oncology, Zhongda Hospital, Medical School of Southeast University, Nanjing, Jiangsu 210009, P.R. China

**Keywords:** Rituximab, microbubble, ultrasound, theranostics, B cell lymphoma

## Abstract

This study evaluated rituximab-conjugated, doxorubicin-loaded microbubbles (RDMs) in combination with ultrasound as molecular imaging agents for early diagnosis of B cell lymphomas, and as a targeted drug delivery system. Rituximab, a monoclonal CD20 antibody, was attached to the surfaces of doxorubicin-loaded microbubbles. RDM binding to B cell lymphoma cells was assessed using immunofluorescence. The cytotoxic effects of RDMs in combination with ultrasound (RDMs+US) were evaluated *in vitro* in CD20+ and CD20– cell lines, and its antitumor activities were assessed in Raji (CD20+) and Jurkat (CD20–) lymphoma cell-grafted mice. RDMs specifically bound to CD20+ cells *in vitro* and *in vivo*. Contrast enhancement was monitored *in vivo* via ultrasound. RDM peak intensities and contrast enhancement durations were higher in Raji than in Jurkat cell-grafted mice (P<0.05). RDMs+US treatment resulted in improved antitumor effects and reduced systemic toxicity in Raji cell-grafted mice compared with other treatments (P<0.05). Our results showed that RDMs+US enhanced tumor targeting, reduced systemic toxicity, and inhibited CD20+ B cell lymphoma growth *in vivo*. Targeted RDMs could be employed as ultrasound molecular imaging agents for early diagnosis, and are an effective targeted drug delivery system in combination with ultrasound for CD20+ B cell malignancy treatment.

## INTRODUCTION

Early diagnosis is pivotal for therapeutic success in many types of cancers. Ultrasound (US) molecular imaging is a novel diagnostic approach for early detection of non-hodgkin lymphoma. Recent studies suggest that targeted microbubbles as US contrast agents (TMUCA) may serve as probes for US molecular imaging. TMUCA would improve diagnostic specificity and allow for disease monitoring in real time. TMUCAs can accumulate and remain at the tumor site for long time periods, and imaging at the molecular level can be acquired using US after TMUCA venous injection [1–3]. US molecular imaging also produces quantitative data, exhibits good temporal resolution, is noninvasive, produces no ionizing radiation, and is relatively inexpensive [4]. Over the past decade, various types of TMUCA have been applied for cell-specific targeting with US molecular imaging *in vivo* [5–10], specifically to assess intravascular inflammation, intravascular thrombosis and tumor blood vessels. For early tumor diagnosis, TMUCAs were conjugated with antibodies specific for tumor cell surface antigens. Previous studies showed that the tumor neovasculature is distorted, with an imperfect basement membrane, and no smooth muscle layer [11]. Permeability was also increased, with wall pores approximately 380–780 nm in diameter [11]. Therefore, TMUCA diameters were adjusted to approximately 500 nm for easy passage through vascular endothelial cells and improved molecular imaging.

Targeted microbubbles are promising tumor-targeting drug delivery systems, although their potential utility as US contrast agents has not yet been studied. Most chemotherapy drugs currently have no targeting capabilities, and act on both diseased and non-diseased sites, leading to low therapeutic indices and severe side effects. A targeted drug delivery system can increase chemotherapy drug accumulation specifically at target sites, while reducing non-target impacts. Moreover, targeted microbubbles are both chemically stable and biodegradable, and exhibit prolonged circulation in the blood, with localized drug release. Tumor-specific ligand-like peptides [12, 13], galactose-conjugated chitosan [14], transferrin [15], folic acid [16–19], and monoclonal antibodies [20–22] have been employed to target microbubbles to tumor cells for the treatment of many cancers. Additionally, the combination of targeted drug-loaded microbubbles with US irradiation permeabilizes cell membranes, enhancing drug uptake by tumor cells, and selectively killing tumor cells without harming normal cells. Therefore, targeted drug-loaded microbubbles have potential use in both targeted drug delivery systems and in combination with US molecular imaging.

We hypothesized that Rituximab-conjugated, doxorubicin (DOX)-loaded microbubbles (RDMs) could serve as effective, biocompatible B cell lymphoma-targeting theranostic agents. The present work evaluated the specific binding potential of RDMs targeting CD20 antigen, a tetraspan membrane receptor overexpressed in B cell malignancies, in lymphoma Raji cells. We also assessed the cytotoxicity and antitumor activity of these RDMs in combination with US irradiation *in vitro* and *in vivo*. Finally, targeted US molecular imaging was explored in Raji and Jurkat cell-grafted mice.

## RESULTS

### RDM characterization

In this study, RDMs targeted the lymphoma B cell CD20 antigen (Figure 1). US triggered DOX release, which was then delivered into lymphoma B cells. RDM morphologies and size distributions were observed via scanning electron microscopy (SEM) (Figure 2A) and transmission electron microscopy (TEM) (Figure 2B), respectively. Mean RDM diameter was 411±125.1 nm (Figure 2C). Fluorescence imaging of RDMs revealed dense green (DyLight488-labeled avidin) and red (DOX) fluorescence with morphologies consistent with those observed via confocal laser scanning microscopy (CLSM) (Figure 3A). Targeting moiety quantities on RDM surfaces were evaluated by detecting RDM suspension fluorescence intensity after conjugation. RDM fluorescence intensity was 72.15% that of the DyLight488-labeled avidin samples (Figure 3B). Due to the high affinity of avidin to biotin, we presumed the same high level of adhesion of biotinylated rituximab to the avidin-conjugated DMs.

**Figure 1:** Illustration of RDM structure, and depiction of antigen-specific, tumor cell targeting drug delivery After RDM attachment to CD 20 antigens on Raji cells, US irradiation triggers DOX release and delivery into cells. DOX, doxorubicin; RDMs, rituximab-conjugated, DOX-loaded microbubbles.

**Figure 2:** Microbubble characterization SEM **A**. and TEM **B**. images of RDMs. RDM size distributions as determined by DLS **C**.

**Figure 3:** Microbubble fluorescence and drug release characterization RDM imaging was performed using CLSM as follows: bright field **Aa**., dylight488-avidin on RDMs (green fluorescence) **Ab**., encapsulated DOX in RDMs (red fluorescence) **Ac**. (scale bar = 25μm). Fluorescence absorbance of RDMs **B**. DMs and free avidin were examined to assess rituximab conjugation efficiency. *In vitro* US-triggered DOX release from DMs and RDMs **C**.

### Drug loading and release

RDMs as a targeted drug delivery system were evaluated via the encapsulation efficiency of DOX. DOX encapsulation efficiency in RDMs was 51.2±2.05%. The release profiles of DOX from RDMs and DMs as triggered by US were also examined. The release profile was described as the percentage of cumulative released DOX as a function of time (Figure 3C). Total DOX released was the same for DMs + US and RDMs + US. The results indicated that DOX was about 50% unloaded after 5 h with sonication and about 90% unloaded after 72 h with sonication. This implied that US could promote DOX release from RDMs and DMs through cavitation.

### Targeted properties of RDMs

To estimate the targeted binding capability of RDMs, the affinity of RDMs to CD20 antigen on Raji cells was determined *in vitro*. RDM attachment to CD20 antigen was greater than that of DMs. CLSM imaging showed large amounts of RDMs (green and red fluorescence) aggregated on Raji cell membranes, demonstrating that rituximab enhanced RDM targeted binding to CD20 antigen. Few DyLight488-labeled avidin-conjugated biotinylated DMs were observed on Raji cell membranes. Competition experiments revealed that RDM targeted binding of Raji cells was reduced as CD20 antigen was blocked following rituximab pre-incubation, as indicated by absence of red and green fluorescent microbubbles. Few RDMs were observed on CD20– CEM cell membranes (Figure 4).

**Figure 4:** *In vitro* RDM targeting to Raji cells CLSM imaging of Raji cells after treatment with targeted RDMs and non-targeted DMs. To visualize microbubble location (green and red fluorescence), Raji cell nuclei were stained with DAPI (blue fluorescence), (scale bar = 10μm). Raji cells targeted by RDMs **A**. Raji cells incubated with DMs **B**. Raji cells blocked with excess rituximab (1 mg/mL) for 2 h before RDM treatment **C**. CEM cells incubated with RDMs as a control **D**.

### Cytotoxicity *in vitro*

The therapeutic efficacies of DOX, DOX + rituximab, DMs + US, RDMs + US, and RDMs + US + rituximab were explored *in vitro*. Raji, Daudi, Jurkat, and CEM cell proliferation inhibition was assessed after treatment for 24, 48 and 72 h. Raji and Daudi cell proliferation inhibition was limited, and was the same for DOX, DOX + Rituximab, DMs + US, and RDMs + US + Rituximab. In contrast, RDM + US inhibited Raji cell proliferation after 24 (35.42±2.16%), 48 (52.32±3.42%), and 72 h (82.74±2.97%) (Figure 5A). RDM + US in Daudi cells also reduced proliferation at 24 (32.84±3.31%), 48 (48.79±2.71%), and 72 h (74.85±3.52%) (Figure 5C). Compared with other treatments, RDM + US effectively inhibited Raji and Daudi cell proliferation (P<0.05). However, in Jurkat and CEM cells, all treatments exhibited similar cytotoxicity (Figure 5B & 5D). RDM + US inhibited proliferation in Raji and Daudi cells more than in Jurkat and CEM cells (P<0.05). We also observed time-dependent cytotoxic effects in all groups. These results demonstrated that US-mediated RDM destruction efficiently inhibited CD20+ lymphoma B cell proliferation.

**Figure 5:** Raji, Daudi, Jurkat and CEM cell growth inhibition Cell proliferation inhibition was measured 24, 48, and 72 h after treatment with DOX, DOX + rituximab, DMs + US, RDMs + US, and RDMs + US + rituximab via CCK8 assay. Data are represented as means ± SD (n=3). *P<0.05 compared with RDM + US.

### Cell apoptosis *in vitro*

Raji, Daudi, Jurkat, and CEM cell apoptosis rates were detected quantitatively by flow cytometry 24, 48 and 72 h after various treatments. Raji and Daudi cell apoptosis rates were comparable following DOX, DOX+ rituximab, DMs + US, and RDMs + US + rituximab treatment, although apoptosis was increased in all groups compared to controls. Importantly, RDMs + US induced higher apoptosis rates than other treatments (Figure 6A & 6C, P<0.05). Jurkat and CEM cell apoptosis rates were similar for DOX, DOX + rituximab, DMs + US, and RDMs + US + rituximab, but higher compared to controls (Figure 6B & 6D). Additionally, RDM + US induced higher apoptosis rates in Raji and Daudi cells as compared to Jurkat and CEM cells (P<0.05). Time-dependent apoptosis rates was detected in all groups (Figure 6). Apoptosis rate measurements were consistent with proliferation inhibition results.

**Figure 6:** Raji, Daudi, Jurkat and CEM cell apoptosis Cell apoptosis was measured 24, 48, and 72 h after treatment with DOX, DOX + rituximab, DMs + US, RDMs + US, and RDMs + US + rituximab by flow cytometry. Data are represented as means ± SD (n=3). *P<0.05 compared with RDM + US.

### Cellular uptake of DOX

Because DOX auto-fluoresces, we detected whether 48 h RDMs + US treatment improved Raji, Daudi, Jurkat, and CEM cell DOX uptake using flow cytometry. DOX intracellular RFI for Raji and Daudi cells was similar following DOX, DOX + rituximab, DMs + US, and RDM + US + rituximab treatment. However, DOX intracellular RFI following RDM + US was higher compared to all other treatments (Figure 7A & 7C, P<0.01). DOX intracellular RFI was also similar following all treatments in Jurkat and CEM cells (Figure 7B & 7D). Additionally, DOX intracellular RFI following RDM + US treatment was higher in Raji and Daudi cells as compared to Jurkat and CEM cells (P<0.01). These results suggest that RDM + US treatment increased DOX transfer into lymphoma B cells more than other treatment groups.

**Figure 7:** DOX relative fluorescence intensity (RFI) in Raji, Daudi, Jurkat and CEM cells Cell RFIs were analyzed 48 h after treatment with DOX, DOX + rituximab, DMs + US, RDMs + US, and RDMs + US + rituximab by flow cytometry. Data are represented as means ± SD (n=3). **P<0.01 compared with RDM + US.

### *In vivo* imaging

Arrival time, time to peak, peak intensity, and duration of contrast enhancement were compared via US imaging between non-targeted DMs and targeted RDMs in Raji and Jurkat cell-grafted mice. In Raji cell-grafted mice, there was no difference between DMs and RDMs for arrival time or time to peak, but peak intensity and duration of contrast enhancement were higher for RDMs (P<0.05). In Jurkat cell-grafted mice, there was no difference between DMs and RDMs in any US measurement (Table 1). Additionally, arrival times and times to peak for targeted RDMs were the same in Raji and Jurkat cell-grafted mice. However, RDM peak intensities and the durations of contrast enhancement were higher in Raji as compared to Jurkat cell-grafted mice (Figure 8, *P<0.05). Targeted RDM (Figure 9C & 9F) and non-targeted DM (Figure 9B & 9E) peak intensity images are shown for Raji and Jurkat cell-grafted mice.

**Table 1:** Four parameters (means ± SD) for DMs and RDMs in Raji and Jurkat cell-grafted mice

Indicators	Arrival time (sec)	Time to peak (sec)	Peak intensity (sec)	Duration of contrasenhancement (min)
Raji cell lymphoma				
DMs	2.71 ± 0.09	17.91 ± 0.62	19.98 ± 0.84*	20.12 ± 0.97*
RDMs	2.75 ± 0.10	17.98 ± 0.56	23.27 ± 1.07	24.27 ± 1.05
Jurkat cell lymphoma				
DMs	2.79 ± 0.07	18.25 ± 0.97	20.06 ± 1.32	20.62 ± 1.05
RDMs	2.82 ± 0.08	18.31 ± 1.12	20.17 ± 1.60*	20.99 ± 1.57*

Paired *t*-test in each group between DMs and RDMs

* P<0.05.

**Figure 8:** RDM arrival time, time to peak, peak intensity, and duration of contrast enhancement in Raji and Jurkat cell-grafted mice RDM arrival times and times to peak were the same in Raji and Jurkat cell-grafted mice. RDM peak intensities and contrast enhancement durations were greater in Raji cell-grafted mice than in Jurkat cell-grafted mice. Data are represented as means ± SD (n=3). *P<0.05, #P>0.05.

**Figure 9:** Contrast-enhanced images of targeted RDMs and non-targeted DMs at time to peak in Raji and Jurkat cell-grafted mice Images of lymphoma before injection **A**. & **D**, non-targeted DMs **B**. & **E**. and targeted RDMs **C**. & **F**. at time to peak were acquired in Raji and Jurkat cell-grafted mice. RDM peak intensities and contrast enhancement durations were higher than those of non-targeted DMs in Raji cell-grafted mice, and were higher in Raji as compared to Jurkat cell-grafted mice.

### *In vivo* antitumor activity

This study used a lymphoma nude mouse model to investigate the antitumor effects of RDMs + US *in vivo*. RDMs + US exhibited the strongest tumor inhibition effect in Raji-cell grafted mice. DMs + US, and RDMs + US + rituximab-treated mice exhibited similarly-reduced Raji cell tumor growth rates compared to controls, and inhibited tumor growth more than treatment with DOX and DOX + rituximab (Figure 10A). DOX and DOX + rituximab only slightly inhibited tumor growth *in vivo*. Similarly, DMs + US, RDMs + US, and RDMs + US + rituximab treatment reduced grafted Jurkat cell tumor growth as compared with DOX and DOX + rituximab. Jurkat cell-grafted mouse treatment with DMs + US, RDMs + US and RDMs + US + rituximab resulted in comparable growth inhibition rates (Figure 10C).

**Figure 10:** Anti-tumor treatment effects in Raji and Jurkat cell-grafted mice Average tumor volumes **A**. and body weights **B**. of Raji cell-grafted mice after treatment with different formulations. Average tumor volumes **C**. and body weights **D**. of Jurkat cell-grafted mice after treatment. Data are represented as means ± SD (n=3). *P<0.05.

To assess the potential systemic toxicity of RDMs + US *in vivo*, nude mouse body weights were periodically examined. Raji and Jurkat cell-grafted mice treated with DOX and DOX + rituximab exhibited slow, continuous weight loss beginning on day 8. In contrast both Raji and Jurkat cell-grafted mouse weights increased gradually with saline, DMs + US, RDMs + US, and RDMs + US + rituximab treatments (Figure 10B & 10D). This suggests that DOX treatment caused severe systemic toxicity in nude mice.

TUNEL staining was used to evaluate apoptosis in Raji and Jurkat cell tumors. Sparse apoptosis (green fluorescence) in Raji and Jurkat lymphoma tissues was observed in mice treated with DOX and DOX + rituximab. Raji cell-grafted mouse tissues treated with DMs + US, and RDMs + US + rituximab showed moderate apoptosis, while RDMs + US treatment induced the most apoptosis. Jurkat cell-grafted mouse tissues treated with DMs + US, RDMs + US, and RDMs + US + rituximab showed moderate cell apoptosis. We observed that RDMs + US induced greater apoptosis levels in Raji as compared to Jurkat cell-grafted mice (Figure 11). These results confirmed that RDMs + US could inhibit lymphoma cell growth by inducing apoptosis.

**Figure 11:** TUNEL staining of Raji and Jurkat lymphomas treated with different formulations Raji and Jurkat cell-grafted mice were treated with saline, DOX, DOX + rituximab, DMs + US, RDMs + US, and RDMs + US + rituximab for 21 days. Green: apoptotic cell DNA; Blue: cell nuclei. Scale bar: 10μm.

## DISCUSSION

Microbubble-based targeted drug delivery has been widely investigated as an anti-tumor therapy in combination with US irradiation [23, 24]. Most targeted drug delivery systems exhibit high therapeutic efficacies *in vitro* and *in vivo*. However, few studies have assessed their potential roles, and the roles of microbubbles, in ultrasonic molecular imaging for diagnosis.

In the present work, we conjugated rituximab to DMs (RDMs) to construct TMUCA. We investigated the potential benefits of TMUCA in both US molecular imaging and targeted anti-lymphoma treatment. DMs encapsulated rituximab with 51.2% efficiency, similar to a previous study [25]. The results of US-mediated drug release assays implied that US induced DMs to release DOX in a controlled manner, probably due to cavitation. RDMs effectively targeted the CD20 antigen on lymphoma B cells. Very few non-targeting DMs were observed on or near Raji cells due to the absence of rituximab. Competition experiments indicated that RDM-Raji cell targeting was reduced when CD20 was blocked by rituximab pre-treatment. These results indicate that rituximab conjugation greatly improved DM-lymphoma cell targeting.

In Jurkat and CEM cells *in vitro*, DMs + US, RDMs + US, and RDMs + US + rituximab treatment induced similar levels of cytotoxicity compared to DOX and DOX + rituximab. This verified that US-triggered drug release from the microbubbles was highly efficient. However, RDMs + US treatment inhibited Raji and Daudi cell proliferation most effectively, in agreement with cell apoptosis assay and intracellular DOX RFI results, as well as the results of a previous report [26]. Additionally, another group reported that anti-CD20 nanoparticles carrying hydroxychloroquine and chlorambucil showed promise for treatment of Burkitt's lymphoma [27].

US molecular imaging allows for exploration of pathological processes *in vivo* at cellular and molecular levels [28, 29], and will improve cancer diagnosis and treatment options. B7-H3-targeted US molecular imaging can reportedly improve breast cancer diagnostic accuracy [30]. US molecular imaging also provides a tool for imaging at a molecular level to enhance B cell lymphoma early diagnosis. In this study, we performed enhanced-contrast imaging experiments with targeted RDMs in a B cell lymphoma nude mouse model. RDM peak intensities and durations of contrast enhancement were higher compared to non-targeted DMs in Raji cell-grafted mice, while there was no difference between RDMs and DMs in CD20– Jurkat cell-grafted mice. Antigen-antibody binding occurred in Raji cell lymphoma tissues after targeted RDMs passed through vascular endothelial cell gaps, leading to a considerable number of RDMs adhering to CD20-overexpressing Raji cells, and generating more stable and longer-lasting contrast enhancement *in vivo* compared to non-targeted DMs. Moreover, targeted RDMs remain in tissues long term, leading to higher peak intensities and persistent contrast enhancement in CD20+ Raji cell-grafted mice as compared to CD20–Jurkat cell-grafted mice. Thus, peak intensity and duration of contrast enhancement may be useful primary parameters in further investigations of targeted RDMs in CD20+ B cell malignancies.

In this study, DOX and DOX + rituximab only slightly inhibited lymphoma cell growth *in vivo*. This was attributed to the rapid diffusion of DOX into all mouse tissues following intravenous injection, leading to potential toxic side effects, and smaller amounts of DOX at tumor sites. The DOX molecule also has a short half-life *in vivo*, and may be metabolized in the circulation before reaching the tumor [31]. The lower systemic toxicity and enhanced anti-tumor activity of RDMs + US observed via TUNEL staining may result from the following factors: (1) encapsulation effectively protected DOX from quick clearance in the circulation; (2) RDMs passively and actively aggregated at the tumor site; (3) rituximab-CD20 binding contributed to RDM-Raji cell attachment, facilitating interaction between drug-loaded microbubbles and cells, and improving local drug delivery efficiency [32]; (4) sonoporation may have enhanced drug uptake by tumor cells via cell membrane pore formation [33], and; (5) rituximab as a targeted drug induced antibody-dependent, cell-mediated cytotoxicity, reducing systemic side effects. Thus, the synergistic effect of DOX and rituximab in RDMs effectively inhibited tumor growth. Our results show that RDMs + US is a promising anti-B cell lymphoma treatment strategy.

In conclusion, this study indicated that targeted RDMs specifically bound CD20+ B cell lymphomas. RDMs combined with US irradiation enhanced tumor targeting, reduced systemic toxicity, and inhibited B cell lymphoma cell growth *in vivo*. Additionally, targeted RDMs increased peak intensity and contrast enhancement duration compared to non-targeted DMs in CD20+ B cell lymphoma-grafted mice. Our findings show that targeted RDMs could potentially be employed as US molecular imaging agents for early diagnosis, and are an effective targeted drug delivery system in combination with US irradiation for the treatment of CD20+ B cell malignancies.

## MATERIALS AND METHODS

### Materials

Poly(lactic-co-glycolic acid) (PLGA; 50% lactide, 50% glycolide, MW=10,000 Da) was purchased from Shandong Shuyuan Biotechnology Co., Ltd (Shandong, China). Poly(vinyl alcohol) (PVA,87–89%, MW=31,000-50,000) was obtained from Sigma-Aldrich (St Louis, MO, USA). Doxorubicin (DOX) was obtained from Shenzhen Wanle Pharmaceutical Co., Ltd. (Shenzhen, China). EZ-LinkTM Sulfo-LC-Biotinylation kit was purchased from Thermo Fisher Scientific, Inc. (Rockford, USA). Amine-Peg2000-Biotin was purchased from Nanjing Ling Di Ren Chemical Technology Co., Ltd (Nanjing, China). Avidin and dyLight488-labeled avidin were obtained from Wuhan Boster Biotechnology Co., Ltd (Wuhan, China). Rituximab was obtained from Hoffmann-La Roche, Inc (New Jersey, USA). Cell Counting Kit-8, the Annexin V-FITC cell apoptosis detection kit and the TUNEL apoptosis detection kit were purchased from Beyotime Biotechnology Co., Ltd (Shanghai, China). All chemicals were analytical grade and used without further processing.

### DM preparation

PLGA microbubbles incorporating DOX were fabricated via a double US emulsion evaporation procedure. 0.5 g PLGA was fully dissolved in 10 ml of liquid chloroform via agitation. The PLGA solution was then combined with a 5 mg DOX solution (dissolved in 1.0 mL superpure water), and the mixture was emulsified via US for 120 min at 100 w. 1.0 mL span-80 was then added. The vial was degassed and re-perfused with nitrogen with stirring at 23,000 rpm for 5 min to obtain primary emulsified DMs. The primary emulsion was poured into cold PVA (40 ml, 5%) containing 1.0 ml tween-80, and stirred at 21,000 rpm for 30 min at room temperature for the second emulsion. The double emulsion was poured into isopropyl alcohol (40 ml, 2.5%) and mechanically agitated for 180 min at room temperature to volatilize the chloroform. The supernatant was removed after the solution was centrifuged at 4,800 rpm for 5 min. The precipitate was centrifuged again at 1,800 rpm for 5 min, and resuspended in superpure water. The superpure water wash was repeated several times until the supernatant become transparent. Precipites were resuspended a final time in superpure water and stored at 4°C. DMs were sterilized via cobalt 60 (^60^Co) irradiation.

### RDM preparation

Covalent bonding of the activated carboxyl groups on DM surfaces was performed using the 1-ethyl-3-[3-dimethylaminopropyl] carbodiimide hydrochloride (EDC) method in the presence of N-hydroxysuccinimide (NHS). Prepared DMs were resuspended in phosphate-buffered saline (PBS; pH 4.7), and EDC and NHS in an equimolar ratio were added into the suspension. The carboxyl groups were activated for 60 min at room temperature. The supernatant was removed after centrifugation, and the precipitate was resuspended in PBS. Amine-Peg2000-Biotin in MES buffer was added, and the mixture was incubated for 120 min at room temperature to obtain biotinylated DMs. Biotinylated DMs were incubated with avidin or dylight488-labeled avidin (1mg/mL) for 10 min at room temperature. The mixture was then centrifuged three times and resuspended in PBS to remove surplus dylight488-labeled avidin/avidin. Rituximab was biotinylated using the EZ-LinkTM Sulfo-LC-Biotinylatio kit according to the manufacturer's instructions, and was added to the avidin-biotin conjugated DMs and incubated for 10 min. The RDM suspension was rinsed three times and centrifuged to remove surplus biotinylated rituximab.

### RDM characterization

We explored RDM morphologies using SEM (Hitachi S-3400N, Japan) and TEM (Hitachi H-7600, Japan), and determined RDM mean diameters and size distributions via dynamic light scattering (DLS) (Nanosizer-S, Malvern, London, UK). RDMs were alsoobserved using a CLSM (Olympus, FV1000, JAPAN). Rituximab coupling efficiency was determined by measuring dyLight488-labeled avidin solution and biotinylated DMs suspension absorbances with a fluorescence spectrophotometer (Jasco, FP-6500, JAPAN) at a maximum excitation wavelength of 493 nm and maximum emission wavelength of 518 nm. Rituximab quantities on biotinylated DMs (binding efficiency (%)) were calculated as the ratio of the intensity of biotinylated DM to the intensity of the dyLight488-labeled avidin samples.

### Assessment of DOX loading

Drug encapsulation efficiency was assessed by ultraviolet-visible spectrophotometry (Eppendorf, BioSpectrometer, Germany). A DOX solution standard curve was measured. Then, fresh RDMs were centrifuged and collected. The RDMs were destroyed using a 5% hydrochloric acid ethanol solution, and the mixture was centrifuged at 3000 rpm for 5 min. The optical density of the supernatant was determined at an excitation wavelength of 495 nm. Drug encapsulation efficiency was calculated using the following equation:

Encapsulation efficiency = Wa/Wb × 100%

where Wa represents the total amount of drug in the RDMs, and Wb represents the total weight of DOX used in the RDM preparation.

### Drug release assay

To estimate DOX release, RDM suspensions were enclosed in dialysis bags (MWCO: 10,000 Da), which were placed in 50 mL of PBS with shaking at 100 rpm at 37°C. The suspension was then sonicated with ultrasound (power density = 1.2 W/cm^2^, frequency = 1 MHz, duty cycle = 50%) for 60 s. At 0, 2, 4, 8, 10, 20, 30, 48, 60, and 72h, 1 ml of dialysate was extracted and stored at 4°C for analysis. An equal volume of PBS was added to the container to insure a constant volume. The concentration of DOX in the sample was determined using an ultraviolet spectrophotometer. DOX release was depicted as a function of time. The DM suspension was assessed using the same method.

### Cell cultures

Human lymphoma B cell lines Raji (CD20+) and Daudi (CD20+), human lymphoma T cell line Jurkat (CD20–), and human T-acute lymphoblastic leukemia cell line CEM (CD20–), were grown in RPMI-1640 medium with 10% (v/v) fetal bovine serum (FBS, Gibco, Australian origin) and 1% penicillin-streptomycin, and incubated in a humidified atmosphere at 37°C with 5% CO_2_. For all experiments, cells growing in suspension were subcultured by centrifugation at a ratio of 1:4.

### Cell targeting assay

After Raji and CEM cells were anchored in culture dishes with Poly L lysine solution, 50ul targeted RDMs and non-targeted DMs were added into the dishes. Shaking was used to encourage interactions in Raji cell cultures. After 30 min at room temperature, dishes were washed twice with PBS and observed via CLSM. Five dishes were used for each experiment group. Blocking tests were performed by pre-incubating Raji cells with rituximab for 30 min followed by washing to removing excessive rituximab. CD20– CEM cells were employed as a control, and non-specific uptake of RDMs by CEM cells was examined using the same methods.

### Cytotoxicity *in vitro*

Raji, Daudi, Jurkat, and CEM cells were seeded in 96-well plates at 1×10^5^ cells/well in 100 μl of RPMI-1640 medium. Microbubble samples were adjusted to contain equal amounts of DOX. Cells were treated with DOX (0.5 μg/mL final concentration), DOX + rituximab, DMs combined with ultrasound (DMs + US), RDMs combined with ultrasound (RDMs + US) and RDMs + US. Raji cells were pre-incubated with excessive rituximab for 30 min (RDMs + US + rituximab). After 24, 48 and 72 h, the Cell Counting Kit-8 was used to detect viable cells in each treatment group relative to controls.

### Cell apoptosis *in vitro*

Apoptosis (early and late stage) was determined using an Annexin V/propidium iodide apoptosis kit and flow cytometry (BD Biosciences, USA) with Cell Quest software. Raji, Daudi, Jurkat and CEM cells, after various treatments for 24, 48 and 72 h, were rinsed twice with cold PBS and resuspended in 195 μl of binding buffer solution. Cells were stained with 5 μl FITC-labeled Annexin V and 10 μl propidium iodide for 20 min at room temperature in the dark. Cells treated with medium alone were used as a control.

### DOX fluorescence intensity

Treatments were as follows: DOX, DOX + rituximab, DMs + US, RDMs + US, and RDMs + US + rituximab at final DOX concentrations of 0.5 μg/ml. Raji, Daudi, Jurkat, and CEM cells were washed three times with cold PBS after 48 h treatment, centrifuged, and resuspended in 500 μl PBS. Cells treated with medium alone were used as controls. Intracellular DOX retention (red fluorescence) was examined using flow cytometry. Relative fluorescence intensity (RFI) was calculated as: FI_experiment_/FI_control_.

### RDM-enhanced contrast ultrasound imaging *in vivo*

Cells were inoculated subcutaneously into the backs of five nude mice per cell type, with 6×10^7^ Raji cells per mouse and 2×10^7^ Jurkat per mouse. Imaging was performed using an iU22 ultrasound system (Phllips, Netherland) with a 12 MHz ultrasound probe, 0.1 mechanical index and 54% gain. Mice were anesthetized by injecting 10% hydral and fixed to entirely expose the tumor under the ultrasound probe. Non-targeted DMs were injected first for imaging studies in grafted mice. After the expurgation of non-targeted DMs, the same amount of targeted RDMs was injected. The process was monitored continuously by ultrasonography. US contrast data were quantified with PHILIPS QLab 8.1 software. The arrival time, time to peak, peak intensity, and duration of contrast enhancement were determined. The Animal Ethics Commitment of the Southeast University approved all animal experiments.

### *In vivo* antitumor activity

Raji and Jurkat cell-grafted mice were established additionally as described above. When lymphoma volume reached approximately 100 mm^3^, Raji and Jurkat cell-grafted mice were randomly divided into 6 groups (five mice per group), respectively : control group (saline), DOX, DOX + rituximab, DMs + US, RDMs + US, and RDMs + US + rituximab. Each mouse was treated with the appropriate formulation (3 mg/kg) three times per week. Lymphoma sizes in all mice were examined via digital caliper, and calculated using the equation: V_tumor_ = LW^2^/2 (L: tumor length, W: tumor width). Lymphoma volumes and mouse body weights were determined before every injection. After 21 d of treatment, all mice were sacrificed. Lymphomas were extracted and fixed with 4% paraformaldehyde. To detect cell apoptosis in lymphoma tissues, tissues were sliced into thin sections and stained with a TUNEL apoptosis detection kit. Samples were then stained with DAPI to visualize cell nuclei under a CLSM.

### Statistical analysis

All experiments were performed in triplicate. Data were presented as means ± standard deviation and analyzed using SPSS 16.0 software (SPSS, Chicago, IL, USA). Comparisons were performed using Student's t-test. P<0.05 was considered a significant difference.

## References

[1] Yan F, Xu X, Chen Y, Deng Z, Liu H, Xu J, Zhou J, Tan G, Wu J, Zheng H (2015). A Lipopeptide-Based alphavbeta(3) Integrin-Targeted Ultrasound Contrast Agent for Molecular Imaging of Tumor Angiogenesis. Ultrasound in medicine & biology.

[2] Zhang H, Tam S, Ingham ES, Mahakian LM, Lai CY, Tumbale SK, Teesalu T, Hubbard NE, Borowsky AD, Ferrara KW (2015). Ultrasound molecular imaging of tumor angiogenesis with a neuropilin-1-targeted microbubble. Biomaterials.

[3] Anderson CR, Hu X, Zhang H, Tlaxca J, Decleves AE, Houghtaling R, Sharma K, Lawrence M, Ferrara KW, Rychak JJ (2011). Ultrasound molecular imaging of tumor angiogenesis with an integrin targeted microbubble contrast agent. Investigative radiology.

[4] Chen ZY, Wang YX, Lin Y, Zhang JS, Yang F, Zhou QL, Liao YY (2014). Advance of molecular imaging technology and targeted imaging agent in imaging and therapy. BioMed research international.

[5] Ammirati E, Moroni F, Pedrotti P, Scotti I, Magnoni M, Bozzolo EP, Rimoldi OE, Camici PG (2014). Non-invasive imaging of vascular inflammation. Frontiers in immunology.

[6] Yang H, Xiong X, Zhang L, Wu C, Liu Y (2011). Adhesion of bio-functionalized ultrasound microbubbles to endothelial cells by targeting to vascular cell adhesion molecule-1 under shear flow. International journal of nanomedicine.

[7] Klibanov AL, Rasche PT, Hughes MS, Wojdyla JK, Galen KP, Wible JH, Brandenburger GH (2004). Detection of individual microbubbles of ultrasound contrast agents: imaging of free-floating and targeted bubbles. Investigative radiology.

[8] Hernot S, Unnikrishnan S, Du Z, Shevchenko T, Cosyns B, Broisat A, Toczek J, Caveliers V, Muyldermans S, Lahoutte T, Klibanov AL, Devoogdt N (2012). Nanobody-coupled microbubbles as novel molecular tracer. Journal of controlled release.

[9] van Rooij T, Daeichin V, Skachkov I, de Jong N, Kooiman K (2015). Targeted ultrasound contrast agents for ultrasound molecular imaging and therapy. International journal of hyperthermia.

[10] Baetke SC, Rix A, Tranquart F, Schneider R, Lammers T, Kiessling F, Lederle W (2016). Squamous Cell Carcinoma Xenografts: Use of VEGFR2-targeted Microbubbles for Combined Functional and Molecular US to Monitor Antiangiogenic Therapy Effects. Radiology.

[11] Wang L, Li L, Guo Y, Tong H, Fan X, Ding J, Huang H (2013). Construction and in vitro/in vivo targeting of PSMA-targeted nanoscale microbubbles in prostate cancer. The Prostate.

[12] Fan CH, Ting CY, Liu HL, Huang CY, Hsieh HY, Yen TC, Wei KC, Yeh CK (2013). Antiangiogenic-targeting drug-loaded microbubbles combined with focused ultrasound for glioma treatment. Biomaterials.

[13] Wang C, Wang X, Zhong T, Zhao Y, Zhang WQ, Ren W, Huang D, Zhang S, Guo Y, Yao X, Tang YQ, Zhang X, Zhang Q (2015). The antitumor activity of tumor-homing peptide-modified thermosensitive liposomes containing doxorubicin on MCF-7/ADR: in vitro and in vivo. International journal of nanomedicine.

[14] Villa R, Cerroni B, Vigano L, Margheritelli S, Abolafio G, Oddo L, Paradossi G, Zaffaroni N (2013). Targeted doxorubicin delivery by chitosan-galactosylated modified polymer microbubbles to hepatocarcinoma cells. Colloids and surfaces B, Biointerfaces.

[15] Wang W, Zhou F, Ge L, Liu X, Kong F (2012). Transferrin-PEG-PE modified dexamethasone conjugated cationic lipid carrier mediated gene delivery system for tumor-targeted transfection. International journal of nanomedicine.

[16] Xing W, Zhigang W, Bing H, Haitao R, Pan L, Chuanshan X, Yuanyi Z, Ao L (2010). Targeting an ultrasound contrast agent to folate receptors on ovarian cancer cells: feasibility research for ultrasonic molecular imaging of tumor cells. Journal of ultrasound in medicine.

[17] Butt AM, Mohd Amin MC, Katas H (2015). Synergistic effect of pH-responsive folate-functionalized poloxamer 407-TPGS-mixed micelles on targeted delivery of anticancer drugs. International journal of nanomedicine.

[18] Zhang L, Zhu W, Yang C, Guo H, Yu A, Ji J, Gao Y, Sun M, Zhai G (2012). A novel folate-modified self-microemulsifying drug delivery system of curcumin for colon targeting. International journal of nanomedicine.

[19] Shi Y, Su C, Cui W, Li H, Liu L, Feng B, Liu M, Su R, Zhao L (2014). Gefitinib loaded folate decorated bovine serum albumin conjugated carboxymethyl-beta-cyclodextrin nanoparticles enhance drug delivery and attenuate autophagy in folate receptor-positive cancer cells. Journal of nanobiotechnology.

[20] Koopaei MN, Dinarvand R, Amini M, Rabbani H, Emami S, Ostad SN, Atyabi F (2011). Docetaxel immunonanocarriers as targeted delivery systems for HER 2-positive tumor cells: preparation, characterization, and cytotoxicity studies. International journal of nanomedicine.

[21] Zhang X, Zheng Y, Wang Z, Huang S, Chen Y, Jiang W, Zhang H, Ding M, Li Q, Xiao X, Luo X, Wang Z, Qi H (2014). Methotrexate-loaded PLGA nanobubbles for ultrasound imaging and Synergistic Targeted therapy of residual tumor during HIFU ablation. Biomaterials.

[22] Yang H, Zhao F, Li Y, Xu M, Li L, Wu C, Miyoshi H, Liu Y (2013). VCAM-1-targeted core/shell nanoparticles for selective adhesion and delivery to endothelial cells with lipopolysaccharide-induced inflammation under shear flow and cellular magnetic resonance imaging in vitro. International journal of nanomedicine.

[23] Pu C, Chang S, Sun J, Zhu S, Liu H, Zhu Y, Wang Z, Xu RX (2014). Ultrasound-mediated destruction of LHRHa-targeted and paclitaxel-loaded lipid microbubbles for the treatment of intraperitoneal ovarian cancer xenografts. Molecular pharmaceutics.

[24] Liu H, Chang S, Sun J, Zhu S, Pu C, Zhu Y, Wang Z, Xu RX (2014). Ultrasound-mediated destruction of LHRHa-targeted and paclitaxel-loaded lipid microbubbles induces proliferation inhibition and apoptosis in ovarian cancer cells. Molecular pharmaceutics.

[25] Niu C, Wang Z, Lu G, Krupka TM, Sun Y, You Y, Song W, Ran H, Li P, Zheng Y (2013). Doxorubicin loaded superparamagnetic PLGA-iron oxide multifunctional microbubbles for dual-mode US/MR imaging and therapy of metastasis in lymph nodes. Biomaterials.

[26] He Z, Huang J, Xu Y, Zhang X, Teng Y, Huang C, Wu Y, Zhang X, Zhang H, Sun W (2015). Co-delivery of cisplatin and paclitaxel by folic acid conjugated amphiphilic PEG-PLGA copolymer nanoparticles for the treatment of non-small lung cancer. Oncotarget.

[27] Mezzaroba N, Zorzet S, Secco E, Biffi S, Tripodo C, Calvaruso M, Mendoza-Maldonado R, Capolla S, Granzotto M, Spretz R, Larsen G, Noriega S, Lucafo M, Mansilla E, Garrovo C, Marin GH (2013). New potential therapeutic approach for the treatment of B-Cell malignancies using chlorambucil/hydroxychloroquine-loaded anti-CD20 nanoparticles. PloS one.

[28] Pan D, Lanza GM, Wickline SA, Caruthers SD (2009). Nanomedicine: perspective and promises with ligand-directed molecular imaging. European journal of radiology.

[29] Weissleder R, Pittet MJ (2008). Imaging in the era of molecular oncology. Nature.

[30] Bachawal SV, Jensen KC, Wilson KE, Tian L, Lutz AM, Willmann JK (2015). Breast Cancer Detection by B7-H3-Targeted Ultrasound Molecular Imaging. Cancer research.

[31] Dhar S, Kolishetti N, Lippard SJ, Farokhzad OC (2011). Targeted delivery of a cisplatin prodrug for safer and more effective prostate cancer therapy in vivo. Proceedings of the National Academy of Sciences of the United States of America.

[32] Yan F, Li X, Jin Q, Jiang C, Zhang Z, Ling T, Qiu B, Zheng H (2011). Therapeutic ultrasonic microbubbles carrying paclitaxel and LyP-1 peptide: preparation, characterization and application to ultrasound-assisted chemotherapy in breast cancer cells. Ultrasound in medicine & biology.

[33] De Cock I, Zagato E, Braeckmans K, Luan Y, de Jong N, De Smedt SC, Lentacker I (2015). Ultrasound and microbubble mediated drug delivery: acoustic pressure as determinant for uptake via membrane pores or endocytosis. Journal of controlled release.

